# Lycorine Displays Potent Antitumor Efficacy in Colon Carcinoma by Targeting STAT3

**DOI:** 10.3389/fphar.2018.00881

**Published:** 2018-08-08

**Authors:** Song Wu, Yuling Qiu, Yingying Shao, Shuangshuang Yin, Rui Wang, Xu Pang, Junhong Ma, Chunze Zhang, Bo Wu, Sangho Koo, Lifeng Han, Yi Zhang, Xiumei Gao, Tao Wang, Haiyang Yu

**Affiliations:** ^1^Tianjin State Key Laboratory of Modern Chinese Medicine, Tianjin University of Traditional Chinese Medicine, Tianjin, China; ^2^School of Pharmacy, Tianjin Medical University, Tianjin, China; ^3^Department of Gastrointestinal Surgery, Nankai Hospital, Tianjin, China; ^4^Department of Colorectal Surgery, Tianjin Union Medical Center, Tianjin, China; ^5^School of Fundamental Sciences, China Medical University, Shenyang, China; ^6^Department of Chemistry, Myongji University, Seoul, South Korea

**Keywords:** lycorine, STAT3, target, apoptosis, colorectal cancers

## Abstract

Signal transducer and activator of transcription 3 (STAT3) is an attractive therapeutic target for cancer treatment. In this study, we identify lycorine is an effective inhibitor of STAT3, leading to repression of multiple oncogenic processes in colon carcinoma. Lycorine selectively inactivates phospho-STAT3 (Tyr-705), and subsequent molecular docking uncovers that lycorine directly binds to the SH2 domain of STAT3. Consequently, we find that lycorine exhibits anti-proliferative activity and induces cell apoptosis on human colorectal cancer (CRC) *in vitro*. Lycorine induces the activation of the caspase-dependent mitochondrial apoptotic pathway, as indicated by activation of caspase and increase of the ratio of Bax/Bcl-2 and mitochondrial depolarization. Overexpressing STAT3 greatly blocks these effects by lycorine in CRC cells. Finally, lycorine exhibits a potential therapeutic effect in xenograft colorectal tumors by targeting STAT3 without observed toxicity. Taken together, the present study indicates that lycorine acts as a promising inhibitor of STAT3, which blocks tumorigenesis in colon carcinoma.

## Introduction

Signal transducer and activator of transcription 3 (STAT3) is a pivotal basic factor in various signaling pathways and plays critical roles in tumor cell differentiation, proliferation, angiogenesis, metastasis, apoptosis, and immune-evasion (Chai et al., 2016; Johnson et al., 2018). Multiple lines of evidence show that constitutive activation of STAT3 signaling contributes to tumor progression and development in varieties of human cancers, including prostate, colon, liver, breast, lung, ovary, blood, gastric cancer, and melanoma (Yu et al., 2014a; Wang et al., 2018). Interestingly, STAT3, which is continuously activated, has no effect on the growth of non-cancerous cells. Numerous studies have reported that non-cancerous cells are not sensitive to the loss of function or inhibitor of STAT3 (Huang W. et al., 2016; Son et al., 2017). Therefore, STAT3 is considered as a promising target for antitumor drug development.

Colon carcinoma is one of the most frequently diagnosed malignancies worldwide (Siegel et al., 2018). Despite significant advances in early screening, surgery and localized therapeutic intervention, the 5-year survival rate of patients with advanced colon carcinoma is only 8% (Miller et al., 2016; Siegel et al., 2018). There is a severe lack of highly reliable strategies for better clinical prevention/therapy. Therefore, it is urgent to develop novel approaches for the treatment of colon cancer. The STAT3 signaling pathway has been reported to play a key role in colon tumorigenesis, including but not limited to the promotion of cell death during development. STAT3 may be a potential therapeutic target for drug discovery of human colon carcinoma (Siveen et al., 2014; Zhao et al., 2016).

Natural products have gained much attention as a source of therapeutic agents, containing inherently large-scale structural diversity and have been the basis of treatment of human diseases for many years (David et al., 2015; Newman and Cragg, 2016; Buenz et al., 2018). It is normally served as excellent starting points for inhibitor design and development. Previous research reported that some nature products inhibited STAT3 activity via functional interaction such as curcumin, toosendanin, and resveratrol (Liu et al., 2014; Chelsky et al., 2017; Zhang et al., 2017). However, the defined molecular mechanisms of them on STAT3 remain elusive.

In this study, we have demonstrated that lycorine inhibits the growth of CRC by inducing apoptosis *in vitro*. Lycorine induces the activation of the caspase-dependent mitochondrial apoptotic pathway. We identify lycorine is an effective inhibitor of STAT3, leading to repression of multiple oncogenic processes in colon carcinoma. Overexpressing STAT3 greatly blocks these effects by lycorine in CRC cells. Finally, lycorine-induced apoptosis suppresses the growth of xenograft colorectal tumors by targeting STAT3 without remarkable toxicity. Taken together, these results suggest that lycorine serves as a novel drug candidate via targeting STAT3 for future CRC therapy.

## Results

### Lycorine Inhibits Growth and Promotes Apoptosis in CRC Cells

The chemical structure of lycorine is shown in **Figure 1A**. We first evaluated the growth inhibitory effect of lycorine on two typical CRC cell lines (SW480 and RKO). As shown in **Figures 1B–E**, cell viability of CRC cell lines was dramatically decreased by lycorine in dose- and time- dependent manner. Consistently, lycorine reduced clonogenic capacity compared with control cells (**Figures 1F,G**). Furthermore, to explore the apoptosis effect of lycorine on CRC cells, we employed Annexin V staining, and lycorine markedly promoted CRC cells apoptosis (**Figures 1H,I**). Taken together, these results suggest that lycorine suppresses proliferation and induces apoptosis in CRC cells.

**FIGURE 1:** Lycorine inhibits growth and promotes apoptosis in CRC cells. **(A)** Chemical structure of lycorine. **(B–E)** Cell viability was determined using MTT assay in RKO and SW480 cells treated with lycorine at indicated concentrations and time. **(F,G)** The colongenicity of RKO and SW480 cells were determined after treatment with lycorine at indicated concentrations for 10 days. **(H,I)** The percentage of apoptotic cells was determined by Annexin V staining. For **(B–E,H,I)**, data are shown as mean ± SD (*n* = 3); ^∗^*P* < 0.05; ^∗∗^*P* < 0.01 compared with control (Student’s *t*-test).

### Lycorine Promotes CRC Apoptosis Through Caspase-Dependent Pathway

To further investigate the effect of lycorine on apoptosis in CRC cells, Western blot assays and caspase activity detection were performed. In CRC cells, lycorine dramatically increased cleaved caspase-3 and subsequent proteolytic cleavage of PARPs protein levels (**Figures 2A,B**). Moreover, treatment of CRC cells with lycorine led to a marked increase in caspase activity (**Figures 2C,D**). More importantly, pretreatment with ZVAD-FMK, a Pan-caspase inhibitor, largely blocked the effect of lycorine-increased activation of cleaved caspase-3 and PARP proteins (**Figures 2E,F**). Importantly, ZVAD-FMK treatment also significantly abolished the effect of lycorine-regulated cell viability (**Figures 2G,H**). Collectively, these results suggest that lycorine triggers apoptosis via caspase-dependent pathway in CRC cells.

**FIGURE 2:** Lycorine promotes CRC apoptosis via caspase-dependent pathway. **(A,B)** RKO and SW480 cells were treated with indicated concentrations of lycorine for 48 h. The protein levels of Cleaved caspase3 and PARP were detected by Western blot assays. **(C,D)** Activity of caspase-3 was evaluated by caspase colorimetric assays. **(E–H)** RKO and SW480 cells were treated with lycorine with and without Z-VAD-FMK respectively. **(E,F)** The levels of cleaved caspase-3 and PARP proteins were determined by Western blot assays. **(G,H)** Cell viability was measured by MTT assay. For **(C,D)**, data are shown as mean ± SD (*n* = 3); ^∗^*P* < 0.05; ^∗∗^*P* < 0.01 compared with control (Student’s *t*-test). For **(G,H)**, data are shown as mean ± SD (*n* = 3); ^∗∗^*P* < 0.01 compared with control; ^##^*P* < 0.01 compared with control cells treated with lycorine (Student’s *t*-test). All the western data shown are representative of at least three independent experiments.

### Lycorine Promotes CRC Apoptosis via the Mitochondrial Pathway

Mitochondrial pathway is one of the major pathways mediating cell apoptosis. In order to determine whether lycorine-induced apoptosis on CRC cells was via the mitochondrial pathway, expression of major regulators of mitochondrial apoptosis and mitochondria membrane depolarization were detected. As indicated in **Figures 3A,B**, after exposure to lycorine, CRC cells showed an up-regulation of Bax and a down-regulation of Bcl-2, which led to a dose-dependent increase of the ratio of Bax/Bcl-2, and an increased cell proportion of depolarized mitochondria after being treated with lycorine (**Figure 3C**). Subsequently, knocking down Bax using siRNA significantly attenuated the effect of lycorine-induced cell death (**Figures 3D–F**). These data further indicate that lycorine-induced apoptosis is mediated by the mitochondrial pathway.

**FIGURE 3:** Lycorine promotes CRC apoptosis via the mitochondrial pathway. **(A)** Western blotting analysis shows that the protein expression of Bcl-2 and Bax was measured in RKO and SW480 cells treated with indicated concentrations of lycorine for 48 h. **(B)** Density ratios of Bax/Bcl-2 protein expression level were shown in the histogram. **(C)** The membrane depolarization of mitochondria was detected by flow cytometer. **(D)** Bax in RKO and SW480 cells was transiently transfected with two individual Bax siRNA (si.Bax-1 and si.Bax-2) or control siRNA (si.Control) for 48 h and was determined by Real-time PCR and Western blot assays. **(E)** Cell viability was determined in lycorine-inhibited and Bax-knocked down RKO and SW480 cells for 48 h. For **(B–D)**, data are shown as mean ± SD (*n* = 3); ^∗^*P* < 0.05; ^∗∗^*P* < 0.01 compared with control (Student’s *t*-test). For **(E**,**F)**, data are shown as mean ± SD (*n* = 3); ^∗∗^*P* < 0.01 compared with control; ^##^*P* < 0.01 compared with si.control transfected cells treated with lycorine (Student’s *t*-test). All the western data shown are representative of at least three independent experiments.

### Lycorine Targets STAT3 in CRC Cells

In previous studies, we have found that lycorine markedly induced autophagy and apoptosis via TCRP1/Akt/mTOR axis inactivation in human liver cancer cells. It is not clear whether the same pathway was also triggered in colon cancer cells. As shown in **Supplementary Figures 1A,B**, lycorine treatment did not significantly affect the protein expression of TCRP1 in colon cancer cells. To investigate whether STAT3 is a direct target of lycorine, CETSAs were performed to demonstrate the direct binding between STAT3 protein and lycorine in *cellulo*. As shown in **Figures 4A,B**, lycorine treatment significantly inhibited STAT3 protein degradation compared with control. Furthermore, to determine whether lycorine could physically interact with STAT3, the pull-down assays were performed. As shown in **Figure 4C**, STAT3 was successfully pulled down by lycorine-conjugated beads compared with the vehicle control beads, indicating that there was a direct binding between STAT3 and lycorine inside cells. In order to identify the potential active sites of lycorine to STAT3, molecular docking experiments were conducted between lycorine and the crystal structure of STAT3 (PDB code: 1BG1) by using Discovery Studio 2017 R2. CDOCKER experiments revealed the best pose of ligand and the actual binding mode of ligand in 3D. To simulating the phosphorylation of STAT3’s 705 site, the modeling sequence modified the TYR residue to PTR. These results indicate that lycorine could enter into the SH2 domain active site of STAT3 and stay in the binding pocket surrounded by key residues (PRT705, Pro695, Pro704, and Gln692). It is worth noting that lycorine can bind to the 705 site after mutation, revealing the reason why STAT3 activity was successfully blocked (**Figures 4D–F**).

**FIGURE 4:** Lycorine targets STAT3 in CRC Cells. **(A,B)** cells were treated with 40 μM of lycorine for 24 h and subsequently heated at different temperature for 3 min. after freeze-thaw cycles for cell lysis, the soluble STAT3 protein levels bound to a drug were visualized by Western blot assays. **(C)** Pull-down assay showing an interaction between lycorine and STAT3. Lycorine was conjugated with epoxy-activated Sepharose 6B. **(D–F)** Docking model of lycorine with STAT3. **(D)** The interaction pattern of lycorine with the residues. **(E)** Lycorine binding with the pocket is composed of hydrogen bonds. **(F)** 2D diagram between the receptor and ligand. All the western data shown are representative of at least three independent experiments.

### Lycorine Promotes Caspase-Dependent Mitochondrial Apoptosis via STAT3 Inactivation

To further determine the STAT3 inhibitory effect, we detected the constitutive activation of STAT3 in CRC cells using a specific antibody against phospho-STAT3 (Tyr-705). As shown in **Figures 5A,B**, lycorine markedly downregulated the phosphorylation level of STAT3 (Tyr-705), but there was no noticeable difference in its total expression in CRC cells. Next, we found that ectopic STAT3 expression in CRC cells dramatically blocked lycorine-induced apoptosis related protein expressions. And ectopic STAT3 expression in CRC cells clearly suppressed lycorine-induced Bax, cleavage of caspase-3 and cleavage of PARP, and also blocked lycorine-inhibited Bcl-2 protein expression (**Figure 5C**). In addition, STAT3 overexpression dramatically blocked the inhibitory effect of lycorine on colony formation and cell viability (**Figures 5D–F**). Furthermore, pretreatment of LY294002 enhanced the conversion of LC-3B, cleavage of caspase-3 and cleavage of PARP, and blocked the expression of p62 induced by lycorine (**Figure 5C**). Furthermore, combination of lycorine with stattic further promoted cell death in CRC cells compared with lycorine treatment alone (**Supplementary Figures 1C,D**). Collectively, these results suggest that lycorine induced the activation of the caspase-dependent mitochondrial apoptotic pathway through targeting STAT3 *in vitro*.

**FIGURE 5:** Lycorine promotes caspase-dependent mitochondrial apoptosis via STAT3 inactivation. **(A**,**B)** RKO and SW480 cells were treated with indicated concentrations of lycorine for 48 h. The protein levels of p-STAT3 were determined by Western blot assays. Total STAT3 expressions were detected as the internal control. **(C–E)** Cells transfected with STAT3 (STAT3 Vec) or empty vector (Control Vec) followed by lycorine treatment. **(C)** The protein levels of p-STAT3, STAT3, PARP, cleaved caspase-3, Bax, and Bcl-2 were detected by Western blot assays. **(D)** The colony formation capability was detected by colonogenic assay. **(E)** The cell viability was measured by MTT assay. For **(E,F)**, data are shown as mean ± SD (*n* = 3); ^∗∗^*P* < 0.01 compared with Vector control; ^##^*P* < 0.01 compared with Vector control transfected cells treated with lycorine (Student’s *t*-test). All the western data shown are representative of at least three independent experiments.

### Lycorine Blocks Growth and Development in Colorectal SW480 Xenograft Tumors

To investigate whether lycorine blocks CRC growth and development *in vivo*, we established a colon tumor xenograft nude mice model by injecting human SW480 cells. As shown in **Figure 6A**, macroscopically, the size of lycorine-treated tumors was significantly decreased compared with that of the control group. Consistently, tumor weight in lycorine-treated mice was much less than that of the control group (**Figure 6B**). There was no noticeable change in body weight between the control and lycorine-treated groups (**Figure 6C**). Xenografts treated with lycorine had an obviously decreased growth rate as compared with those treated with control (**Figure 6D**). Furthermore, Western blot and IHC staining were conducted in CRC xenograft tumors. As shown in **Figure 6E**, lycorine treatment dramatically increased cleaved caspase-3 and PARPs, and decreased Bcl-2 protein expression in SW480 tumors compared with that of the control group. Consistently, lycorine treatment exhibited much higher positive staining of cleaved caspase-3 and PARP than that of the control group (**Figure 6F**). More importantly, lycorine treatment attenuated the phosphorylation level of STAT3 in SW480 xenograft tumors (**Figure 6G**). Accordingly, IHC staining demonstrated that positive staining of phosphorylated STAT3 was much lower in lycorine-treated xenografts tumors compared with that of the control group (**Figure 6H**). Collectively, our results suggest that STAT3 plays a key role in lycorine-regulated caspase-dependent mitochondrial apoptosis in CRC.

**FIGURE 6:** Lycorine blocks growth and development in colorectal SW480 xenograft tumors. **(A–H)** BALB/c nude mice were inoculated with SW480 cells and treated with lycorine or vehicle. **(A)** Tumors were isolated and photographed. **(B)** Tumors were weighted. **(C)** Bodies were weighted. **(D)** Tumor volumes were measured every 3 days. **(E)** PARP, cleaved caspase-3 and Bcl-2 levels were determined in xenograft tumors by Western blot assays. **(F)** PARP and cleaved caspase-3 expressions were determined by IHC staining in xenograft tumors. **(G)** p-STAT3 and total STAT3 levels were determined in xenograft tumors by Western blot assays. **(H)** p-STAT3 expressions were determined by IHC staining in xenograft tumors. For **(B**,**D)**, data are shown as mean ± SD (*n* = 9). ^∗^*P* < 0.05; ^∗∗^*P* < 0.01 compared with control (Student’s *t*-test). For **(F**,**H)**, representative images were conducted as indicated. ^∗∗∗^*P* < 0.001; Scale bars: 50 μm. All the western data shown are representative of at least three independent experiments.

Taken together, our results suggest that lycorine, blocks tumorigenesis in colon carcinoma, acts as a promising inhibitor of STAT3.

## Discussion

Natural products, as important source of medicine and therapeutics, play a vital role in treatment of human diseases (David et al., 2015; Newman and Cragg, 2016). Lycorine, an active natural compound, has been reported to possess potential anticancer activities (Hu et al., 2015; Jin et al., 2016; Roy et al., 2016; Wang et al., 2017; Yu et al., 2017). However, the defined molecular basis of lycorine on CRC remains unveiled. In this study, we have for the first time demonstrated that lycorine induces the activation of the caspase-dependent mitochondrial apoptotic pathway via targeting STAT3, leading to the repression of the growth of CRCs *in vitro* and *in vivo*.

Apoptosis, as a kind of programmed cell death, is a highly controlled and tightly regulated process involving a number of energy-dependently molecular and biochemical events (Berchtold and Villalobo, 2014; Fuchs and Steller, 2015). Apoptosis is usually occurred in the mechanism of mitochondrial pathway or death receptor pathway, or both at the same time (Mariño et al., 2014; Flusberg and Sorger, 2015). In mitochondrial pathway, mitochondrial transmembrane potential and Bcl-2 family proteins are widely involved (Mariño et al., 2014; Roy et al., 2014; Hata et al., 2015). Numerous anticancer drug leads exhibit pro-apoptosis activity via mitochondrial pathway. We have found that lycorine initiates apoptotic cell death in CRC cells, which is supported by the result of V-FITC/PI double staining. We also have found that upregulation of Bax, downregulation of Bcl-2, increased ratio of Bax/Bcl-2 as well as mitochondrial depolarization are observed 48 h after lycorine treatment. Furthermore, knockdown of ectopic Bax by siRNA largely abolished lycorine-induced proapoptotic effect in CRC cells. Caspases which belong to the family of cysteine proteases are integral components of the apoptotic pathway. Recently, many studies have shown that a variety of chemotherapeutic agents promote apoptosis through the activation of caspases (Roy et al., 2014; Fulda, 2015; Hata et al., 2015). In this study, we have found that lycorine treatment markedly augments caspase activity, and upregulates cleaved caspase-3 and PARP. Furthermore, blocking the caspase pathway largely abolishes the apoptotic effect of lycorine. Together, these results suggest that lycorine induces caspase-dependent apoptosis via mitochondrial pathway in CRC cells.

Interestingly, we have investigated not only the classical hub proteins such as caspases and Bcl-2 family that can be activated the main apoptotic pathways, but also STAT3, a ‘novel’ hub protein/target, has been found in core apoptotic pathways. Previous study has shown that STAT3 dimerization is blocked and complex formation of STAT3 is impaired by Toosendanin, a triterpenoid saponin compound, which can inhibit osteosarcoma growth and metastasis (Zhang et al., 2017). In addition, other study has reported that Erasin promotes apoptosis in Erlotinib-resistant lung cancer cells by direct inhibition of tyrosine phosphorylation of STAT3 (Lis et al., 2017). Moreover, a recent study has demonstrated that S3I-201.1066, a novel small-molecule, binds with a high affinity to STAT3, disrupts STAT3 activation and function, and thereby increases anti-breast cancer activity *in vitro* and *in vivo* (Zhang et al., 2010; Yeh and Frank, 2016). Inhibitors directly interact with the STAT3 protein can be distinguished based on the distinct binding domain. STAT3 proteins contain three major domains: the coiled-coiled domain at the N terminus, the DNA-binding domain, and the SH2 transactivation domain at the C terminus (Wake and Watson, 2015; Chai et al., 2016). The SH2 domain of STAT3 is responsible for upstream receptor kinases recognition and the dimerization that is involved in DNA binding and gene expression, and it is considered to be the most promising targetable site for STAT3 (Namanja et al., 2016; Genini et al., 2017; Huang et al., 2018). Drugs targeting the SH2 domain could inhibit phosphorylation at tyrosine residue 705 (Tyr-705), which prevents tyrosine phosphorylation of Stat monomers, nuclear translocation, and target gene expression, and thus promotes apoptosis (Furtek et al., 2016; Spitzner et al., 2018).

In the present study, we find direct binding between STAT3 and lycorine by pull-down and CETSAs. Moreover, we found that lycorine selectively inactivates phospho-STAT3 (Tyr-705) and directly binds to the SH2 domain of STAT3 by molecular docking. The inhibition effects are further confirmed by Western blot: lycorine dramatically inhibits phospho-STAT3 (Tyr-705) in a dose dependent manner, but there is no obvious change in its total expression in CRC cells. Furthermore, we find that ectopic STAT3 expression markedly blocks lycorine-regulated mitochondrial apoptosis and anti-proliferative activity in CRC cells.

In addition, we have found that lycorine inhibits tumor growth in SW480 xenograft model without marked toxicity. Moreover, IHC staining and Western blot demonstrates that lycorine treatment leads to the active levels of cleaved caspase-3 and subsequent proteolytic cleavage of PARPs in xenografted tumors. More importantly, the levels of p-STAT3 also are inhibited by lycorine compared with control, indicating that the anti-tumor activity of lycorine is against colon cancer cells in xenograft tumors by STAT3-regulated apoptosis manners.

In summary, this study demonstrates that lycorine induces the activation of the caspase-dependent mitochondrial apoptotic pathway through targeting STAT3, which in turn inhibits the tumor growth of CRC, and the present study indicates that lycorine acts as a promising candidate that blocks tumorigenesis in colon carcinoma.

## Materials and Methods

### Cell Culture and Cell Treatments

Human CRC cell lines SW480 and RKO cell were obtained from ATCC in April 2017. The used cells were resuscitated within 1 month. The cell lines were identified by PCR-amplified short tandem repeat analysis. Mycoplasma contamination was excluded in these cell lines. Cells were maintained at 37°C in DMEM supplemented with 10% FBS and 1% penicillin/streptomycin in a humidified atmosphere with 5% CO_2_. Expression vector of human STAT3 was designed and purchased from Servicebio Technologies (Wuhan, China). For siRNA knockdown, siRNA oligos against Bax was purchased respectively from GenePharma (Shanghai, China). Lycorine (purity > 98%) was purchased from Shanghai Yuanye Bio-Technology (Shanghai, China). A 20 mM stock solution was prepared in dimethyl sulfoxide (DMSO), and stored in aliquots at −20°C. Z-VAD-FMK was obtained from Calbiochem (San Diego, CA, United States). MTT [3-(4, 5-dimethyl-2-thiazolyl)-2, 5-diphenyl-2-H-tetrazolium bromide] reagent was purchased from Sigma-Aldrich (St. Louis, MO, United States).

### Cell Viability Assay

Cell viability was determined by MTT assay. In brief, Human CRC cells (5 × 10^3^ cells/well) were treated with lycorine at indicated concentrations and time, and MTT solution was added and incubated for 4 h at 37°C. Then, medium was removed. 100 μl DMSO was added and absorbance at 570 nm was determined by microplate reader. For blocking study, cells were pre-incubated with 50 μM Z-VAD-FMK for 1 h, and then treated with lycorine (40 μM) for 48 h.

### Measurement of Mitochondrial Membrane Potential (MMP)

Mitochondrial membrane potential (MMP) in Human CRC cells treated with lycorine at the indicated concentrations for 48 h was measured by flow cytometry with JC-1, a dual-emission fluorescent dye. There are two excitation wavelengths, 527 nm (green) for the monomer form and 590 nm (red) for the J-aggregate form. The cells were harvested and incubated with 10 μM JC-1 for 30 min at 37°C. The cells were analyzed by a flow cytometer (Becton Dickinson).

### Assay for Annexin V Staining

Apoptosis was measured by staining cells using Muse^TM^Annexin V & Dead Cell Assay Kit (Millipore, Billerica, MA, United States), and cells were analyzed in a bench Muse Cell Analyzer (Millipore, Billerica, MA, United States) according to manufacturer’s instructions.

### Quantitative Real-Time PCR

Total RNA was purified as described above (Huang H. et al., 2016). The primers for Bax were purchased from Sangon Biotech. Real-time PCR was done in triplicate with SYBGreen PCR mixture (Applied Biosystems, Foster City, CA, United States). The expression of genes was normalized to the *Actin* gene. The primers used for quantitative real-time PCR were as follows: for *Bax*, 5′-GGAATTCTGACGGCAACTTCAACTGGG-3′ and 5′-GGAATTCTTCCAGA TGGTGAGCGAGG-3′; For *Actin*, 5′-GGACTTCGAGCAAGAGATGG-3′ and 5′-AGCACTGTGTTGGCGTACAG-3′.

### Colony Formation Assay

Colony formation assay was determined as previously described (Yu et al., 2017). Human CRC cells were seeded into 6-well plates and incubated overnight. Cells were then treated with lycorine at the indicated concentrations for 48 h. After being rinsed with fresh medium, the colonies were formed, fixed with 4% paraformaldehyde, stained with 0.1% crystal violet, and then counted in indicated time periods.

### Xenograft Tumorigenicity Assays

SW480 Cells (5 × 10^6^ in 0.2 mL PBS) were inoculated (*via* s.c. injection) into 7-week-old BALB/c female athymic nude mice (Taconic). When tumor volumes reached 100 mm^3^, mice were randomized into two groups (*n* = 9, per group) and received i.p. injection with lycorine (20 mg/kg/day) or vehicle every other day for 33 days. Tumor volume and body weight were monitored every 3 days. All animal experiments were conducted under protocols approved by the Animal Care and Use Committee of Tianjin University of Traditional Chinese Medicine (TCM-LAEC20170027). No specific exclusion or inclusion used for animal experiments.

### Immunohistochemistry Assay

Immunohistochemistry (IHC) analysis was conducted as described previously (Yu et al., 2014b). Tissue sections were excised, formalin-fixed, paraffin-embedded, and then incubated with anti-Cleaved caspase-3, anti-PARP and anti-p-STAT3 antibodies overnight at 4°C, followed by biotinylated secondary antibody. Images were visualized by a Leica DM4000B microscope (Leica, Wetzlar, Germany).

### Caspase Colorimetric Assay

The enzymatic activity of the caspases was assayed using a colorimetric assay kit according to the manufacturer’s protocol (Calbiochem, San Diego, CA, United States). The cells were incubated in the absence and presence of lycorine at indicate concentrations respectively for 48 h, and then the cells were incubated with 50 μl reaction buffer and 5 μl specific colorimetric peptide substrates, Ac-Asp-Glu-Val-Asp (DEVD)-pNA for caspase-3, at 37°C for 1 h in the dark. The absorbance at 405 nm was determined by measuring the changes with an ELISA reader.

### Western Blot Assays

Standard Western-blot assays were analyzed as conducted as previously described (Huang H. et al., 2016; Yu et al., 2017). Antibodies against phospho-STAT3 (Tyr-705), total STAT3 and Cleaved caspase-3 (D175) were purchased from Cell Signaling Technology (Danvers, MA, United States). Anti-PARP1/2 (H250), Bax (SC-493), and Bcl-2 (SC-7382) antibodies were purchased from Santa Cruz Biotechnology (Santa Cruz, CA, United States). Anti-β-actin (A5441) antibody was purchased from Sigma-Aldrich (St. Louis, MO, United States).

### Cellular Thermal Shift Assays

Cellular thermal shift assays (CETSAs) were conducted to determine the direct binding between lycorine and STAT3 in cellular. Briefly, cells were pretreated with DMSO or lycorine (40 mM) for 48 h, chilled on ice, washed with PBS plus protease inhibitor cocktail and then transferred into 200 ml PCR tubes and heated for 3 min at indicated temperature. Subsequently, cells were lysed using liquid nitrogen and two repeated cycles of freeze-thaw. Precipitated proteins were separated from the soluble fraction at 20,000 *g* for 20 min at 4°C to clarify, soluble proteins, collected in the supernatant, were kept at −80°C until Western blot assays.

### Pull-Down Assay

Lycorine (1 mg) was dissolved in 1 mL of coupling buffer (0.1 M NaHCO_3_, pH 11.0 containing 0.5 M NaCl) and conjugated with epoxy-activated Sepharose 6B. The epoxy-activated Sepharose 6B was swelled and washed in distilled water on a sintered-glass filter and then washed with the coupling buffer. The epoxy-activated Sepharose 6B beads were added to the lycorine-containing coupling buffer and rotated at 4°C overnight. After washing, unoccupied binding sites were blocked with 0.1 M Tris-HCl (pH 8.0) for 2 h at room temperature. The lycorine-conjugated Sepharose 6B was washed with three cycles of alternating pH wash buffers (buffer 1: 0.1 M acetate and 0.5 M NaCl, pH 4.0; buffer 2: 0.1 M Tris-HCl and 0.5 M NaCl, pH 8.0). The control unconjugated epoxy-activated Sepharose 6B beads were prepared as previously described in the absence of lycorine. The cell lysate was mixed with lycorine-conjugated Sepharose 6B or with Sepharose 6B at 4°C overnight. The beads were then washed three times with TBST. The bound proteins were eluted with SDS loading buffer. The proteins were resolved by SDS-PAGE followed by immunoblotting with an antibody against STAT3.

### Molecular Docking

Docking simulations were carried out with Discovery Studio 2017 R2. Three dimensional structures of lycorine were downloaded from PubChem Compound^1^. The structure of STAT3 (PDB code: 1BG1) was obtained from the protein data bank^2^. Receptor preparation includes removing water molecules and impurity ions and adding polar hydrogen atoms. The predicted binding energy (kcal mol^−1^) was calculated. The most reasonable complex structures were identified according to binding energy and selected as initial models for the subsequent simulations. Docking of ligand and receptor to CDOCKER Experiment using software Discovery Studio 2017 R2. Select the highest scoring ligand receptor binding pose and obtain the RMSD.

### Statistical Analysis

Data were presented as mean ± SD of at least three independent experiments. The statistical differences in xenograft tumor growth in response to lycorine treatment were analyzed by one- or two-way ANOVA, followed by Student’s *t*-test. All other *P*-values were performed by a two-tailed Student’s *t*-test with Welch’s correction (assume unequal variance). The correlation between two factors was evaluated by correlation analysis, and Spearman correlation coefficients were calculated to estimate the correlations. The statistically variation (*P* < 0.05) was considered to be significant.

## Author Contributions

TW and HY contributed to conception and design. SW, YQ, YS, SY, RW, XP, JM, CZ, and BW performed the experiments. YQ, SK, LH, YZ, XG, TW, and HY analyzed the data. YQ and HY wrote the manuscript.

## Conflict of Interest Statement

The authors declare that the research was conducted in the absence of any commercial or financial relationships that could be construed as a potential conflict of interest.

## Footnotes

1 http://pubchem.ncbi.nlm.nih.gov

2 http://www.rcsb.org/pdb
